# In Search of a Neurotologic Profile in COVID-19 — A Study in Health Care Workers

**DOI:** 10.7759/cureus.21015

**Published:** 2022-01-07

**Authors:** Alejandra Espinoza-Valdez, Erika Celis-Aguilar, Francelia Torres-Gerardo, Natalia Cantú-Cavazos, Edgar Dehesa-Lopez

**Affiliations:** 1 Otolaryngology - Head and Neck Surgery, Universidad Autonoma de Sinaloa, Culiacan, MEX; 2 Statistics, Universidad Autonoma de Sinaloa, Culiacan, MEX

**Keywords:** covid-19, sars-cov-2, vestibular diseases, otolaryngologic diseases, ear diseases

## Abstract

Introduction

COVID-19 is an emerging disease and the neurotologic symptoms are still not well understood. Furthermore, the development of a neurotological profile and its associated factors can help the clinician in the diagnosis and treatment of this disease. The objective is to determine the neurotologic manifestations experienced by COVID-19 positive health care workers and their associated factors.

Methods

A symptoms survey was administered to health care workers who were positive to COVID-19 from September to October 2020. An informed consent form was digitally signed and Google Forms software was used for the survey. Frequencies and percentages were used for categorical variables, and associated clinical features were reported with odds ratios.

Results

We included 209 COVID-19 positive health care workers, 55.5% (n = 116) were women, and 44.5% (n = 93) were men. Fifty-three percent of patients were 20 to 30 years old and 56.4% had at least one comorbidity. The prevalence of neurotological manifestations was 18.6% (n = 39/209), the most frequent symptoms were vertigo (61.5%, n = 24/39), tinnitus (43.5%, n = 17/39), imbalance (43.5%, n = 17/39), and one case of facial paralysis (2.5%, n = 1/39). Neurotological manifestations were associated predominantly with asthenia (*p *= 0.021), loss of smell (*p *= 0.002) and taste dysfunction (*p *= 0.002).

Conclusion

The most common neurotological manifestations were vertigo, tinnitus and imbalance. Clinical features associated with a neurotologic profile were asthenia, hyposmia and dysgeusia.

## Introduction

A new species of coronavirus caused an epidemic outbreak of atypical pneumonias in late December 2019 in Wuhan, China, becoming rapidly a global health problem [1]. SARS-CoV-2 infection (Severe Acute Respiratory Syndrome Coronavirus 2) affects the central nervous and peripheral nervous systems, and muscle; these neurogenic properties explain many of the coronavirus manifestations [2].

Additionally, histologic studies have confirmed the capacity of SARS CoV-2 virus to infect the nervous system. Reverse transcription-polymerase chain reaction (RT-PCR) has detected SARS-CoV genomic sequences in cerebral spinal fluid and brain tissue specimens, also edema and focal degeneration of neurons have been observed in the brains of SARS CoV-2 autopsies [2, 3].

Coronaviruses have both hematogenous and neuro-invasive properties and can produce excitotoxicity, neurodegeneration and apoptosis [4]. Through these mechanisms, they can affect central and peripheral nervous systems. COVID-19 manifestations vary in severity and presentation depending on the genetic and nongenetic factors of the host, among other variables [5].

Currently, there is scant data on neurotological symptoms in COVID-19 positive patients. However, there has been a steady rise in publications with these manifestations in recent literature [6-9]. Regarding the cochlear symptoms of COVID-19, it is possible that COVID-19 could directly damage the cochlear hair cells, thus causing hearing loss [10]. Furthermore, the most frequent neurotological manifestations in COVID-19 patients are tinnitus and, to a lesser extent, vertigo, hearing loss and facial paralysis [6, 11-14].

The objective of this study was to determine the prevalence of neurotological manifestations in COVID-19-positive health care workers and to analyze their association with other clinical symptoms.

## Materials and methods

A descriptive and analytical cross-sectional study was conducted using a survey. The survey was administered through Google Forms from September 15 to October 19, 2020. Information about the otorhinolaryngologic and neurotologic symptoms was obtained from positive SARS-CoV-2 RT-PCR (Reverse Transcriptase - Polymerase Chain Reaction) health care workers.

The version of the survey used is available at figshare [15]. To be included in the study, all participants underwent confirmatory RT-PCR for SARS-COV-2. The survey included 28 sociodemographic questions regarding the participants' occupation, institution, gender, and age, followed by questions on complementary testing (IgG and IgM antigens, chest computed tomography), comorbidities, symptoms and their duration, with an emphasis on otorhinolaryngological and neurotological manifestations. Some questions allowed the selection of multiple answers.

Informed consent was digitally signed by all participants. Data was managed anonymously, as indicated by the Declaration of Helsinki.

For the analysis, the population was divided into two groups: patients with neurotological manifestations, and patients without neurotological manifestations. Patients were classified in the neurotological group if they presented with at least one neurotologic manifestation such as imbalance, vertigo, tinnitus, subjective hearing loss and/or facial paralysis; therefore, some patients had more than one neurotological manifestation.

The results were collected automatically through Google Forms and then transferred to an Excel database for descriptive analysis using Statistical Software for Social Sciences (SPSS, Inc., Version 21, IBM Corp., Armonk, NY, USA). Categorical variables were described as frequencies and percentages, and associations as odds ratios and confidence intervals. A p-value <0.05 was considered statistically significant.

## Results

Sociodemographic data

A total of 209 patients participated in this study, 55.5% (n = 116) were female and 44.5% (n = 93) were male. The most frequent comorbidities were obesity (23.9%, n = 50) and hypertension (14.3%, n = 30).

In the total population, anosmia was present in 45% (n = 94), hyposmia was present in 21% (n = 44), and 34% (n = 71) of participants reported no loss of smell. Regarding dysgeusia, 33% (n = 69) reported ageusia, and 25.4% (n = 53) reported hypogeusia. Other symptoms include otalgia (13.4%), facial pain (11%), and otitis externa (2.4%).

Neurotological manifestations and clinical associations

The prevalence of neurotological manifestations in COVID-19 positive health care workers was 18.6% (n = 39/209).

The neurotological manifestations were vertigo in 61.5% (n = 24/39), tinnitus in 43.5% (n = 17/39), imbalance or unsteadiness (43.5%, n = 17/39), hearing loss (15.3%, n = 6/39) and facial paralysis (2.5%, n = 1/39) (Figure 1).

**Figure 1:** Neurotologic symptoms in COVID-19 positive health care workers.

The group with no neurotologic manifestations had 170 participants and the group with neurotological manifestations had 39 subjects.

There was no difference between baseline demographic variables and neurotologic profile, except for the nursing personnel that showed an increased prevalence of neurotological manifestations (35.9% vs. 11.2%, p = 0.007) (Table 1).

**Table 1:** Baseline demographic characteristics in COVID-19 positive health care workers.

Demographic variables	Total n = 209	Without neurotological manifestations n = 170 n (%)	With neurotological manifestations n = 39 n (%)	p
Gender				0.073
Female	116	89(52.4)	27(69.2)	
Male	93	81(47.6)	12(30.8)	
Age				0.603
20-30 years	111	91(53.5)	20(51.3)	
31-40 years	38	29(17.1)	9(23.1)	
41-50 years	32	27(15.9)	5(12.8)	
51-60 years	21	16(9.4)	5(12.8)	
Over 60 years	7	7(4.1)	0	
Occupation				0.007
Resident (PYG)	58	50(29.4)	8(20.5)	
Medical doctor	63	56(32.9)	7(17.9)	
Nursing personnel	33	19(11.2)	14(35.9)	
Medical students	36	29(17.1)	7(17.9)	
Nurse aide	9	7(4.1)	2(5.1)	
Others	10	9(5.3)	1(2.6)	
Institutions				0.517
Public Institution	179	143(84.1)	36(92.3)	
Private Institution	15	14(8.2)	1(2.6)	
Both Institutions	14	12(7.1)	2(5.1)	
Comorbidities				0.372
Absent	88	74(44.6)	14(35.9)	
Present	117	92(55.4)	25(64.1)	

General manifestations associated with neurotological profile were asthenia (94.9% vs 78.2%, p = 0.021), headache (89.7% vs 72.9%, p = 0.036), and odynophagia (56.4% vs 38.2%, p = 0.047) (Table 2).

**Table 2:** General manifestations in COVID-19 positive health care workers

General clinical manifestations	Total n = 209	Without neurotological manifestations n = 170 n (%)	With neurotological manifestations n = 39 n (%)	p
Asthenia	170	133(78.2)	37(94.9)	0.021
Headache	159	124(72.9)	35(89.7)	0.036
Myalgia	151	123(72.2)	28(71.8)	1.0
Fever	141	119(70)	22(56.4)	0.129
Arthralgia	122	100(58.8)	22(56.4)	0.858
Dry cough	119	95(56.5)	24(61.5)	0.682
Productive cough	12	9(5.4)	3(7.7)	0.682
Diarrhea	98	77(45.3)	21(53.8)	0.376
Odynophagia	88	65(38.2)	22(56.4)	0.047
Dyspnea	87	66(38.8)	21(53.8)	0.105
Anorexia	81	62(36.5)	19(48.7)	0.202
Rhinorrhea	72	59(34.7)	13(33.3)	1.0
Conjunctivitis	33	23(13.5)	10(25.6)	0.086

We found otolaryngologic symptoms associated with a neurotologic profile, such as loss of smell (p = 0.002) and loss of taste (p = 0.002) (Table 3).

**Table 3:** Otolaryngological manifestations in COVID-19 positive health care workers

Otolaryngological manifestations	Total n = 209	Without neurotological manifestations n = 170 n (%)	With neurotological manifestations n = 39 n (%)	p
Otalgia	28	17(10)	11(28.2)	0.005
External otitis	5	3(1.8)	2(5.1)	0.234
Otitis media	1	0	1(2.6)	0.187
Loss of smell	138	104(61.2)	34(87.2)	0.002
Loss of taste	122	91(53.8)	31(81.6)	0.002
Submandibular lymphadenopathy	23	15(11.5)	8(22.2)	0.109
Aphthae	28	24(14.1)	4(10.3)	0.743
Thyroiditis	4	4(2.4)	0	0.596
Xerostomia	93	72(42.4)	21(53.8)	0.214
Facial pain	23	16(9.5)	7(17.9)	0.155

Chest computed tomography (CT) scan was performed in 63.1% (n = 132) of subjects. A total of 44% (n = 92) were CT scan positive for pneumoniae of COVID-19 and 19.1% (n = 40) were CT scan negative for pneumoniae caused by COVID-19. Positive chest CT scan results (n = 92) were significantly associated with the presence of loss of smell (p = 0.001) and loss of taste (p = 0.013). Nevertheless, there was no significant association between the presence of neurotological manifestations and a positive chest CT scan (p = 0.403).

Additionally, patients with hyposmia or anosmia were 4.31 times more likely to present a neurotologic complication, as well as those with dysgeusia were 3.79 times more prone to present neurotologic symptoms (Table 4).

**Table 4:** Variables associated with a neurotologic profile OR: Odds Ratio; CI: Confidence Interval

Variables	OR	95% CI	p
Asthenia	5.14	1.18-22.35	0.021
Loss of smell	4.31	1.606-11.59	0.002
Loss of taste	3.79	1.584-9.098	0.002
Otalgia	3.53	1.49-8.34	0.005
Headache	3.24	1.09-9.63	0.036
Odynophagia	2.09	1.03-4.22	0.047

Treatment

Regarding the treatments used for these patients, 90% (n = 188) reported the use of acetaminophen; azithromycin was used by 66.5% (n = 139) of the participants, ivermectin in 39.2% (n = 82), antivirals 37.3% (n = 78), corticosteroids 35.4% (n = 74), anticoagulants 32.1% (n = 67), steroid inhalers 13.9% (n = 29), hydroxychloroquine 11.5% (n = 24), steroid nebulizers 10% (n = 21), supplemental oxygen 9.6% (n = 20), tocilizumab 7.7% (n = 16) and chlorine dioxide 3.3% (n = 7); 4.3% (n = 9) reported not receiving any treatment.

## Discussion

We present a study that explores neurotological symptoms and their associated clinical variables in a population of health care workers.

Neurotological manifestations

The SARS-CoV-2 can invade the central and peripheral nervous systems, producing in this manner, a wide range of neurological manifestations; from mild symptoms such as loss of smell to others of greater complexity, such as encephalopathy [16-18].

Furthermore, there is a viral neurotropism in SARS-CoV-2 [2]. Direct invasion of the central nervous system by this virus may occur by two routes: hematogenous and via axonal transport. The axonal invasion could lead to the damage of the cranial nerves, for example, the olfactory nerve [19-21].

Our survey described the presence of tinnitus and hearing impairments, similar to previously published studies [14, 22, 23]. Additionally, in our study we found a higher prevalence of vertigo and otalgia [14, 22-24].

Unfortunately, in the literature there are mainly case reports and surveys when reporting for the audio-vestibular assessment of patients with COVID-19 [25], probably due to the contagious nature of the disease, as this precludes more exhaustive research, at least in the beginning of the pandemic, when vaccines were not readily available.

In the study of Viola et al., 38.2% of patients with dizziness had migraine [14]; among our respondents, there was a significant association between headache and neurotological manifestations.

We have reported one case of facial paralysis. This is relevant since current literature suggests that facial paralysis might be the only or the first finding of COVID-19 [12, 13, 26, 27]. Egilmez et al. found in their study that most patients with facial paralysis have a grade 4 on House-Brackmann scale at first admission, and after 2-5 weeks of steroid treatment 37.5% recovered [27].

Other more severe neurological manifestations are encephalitis, Guillain-Barré, cerebrovascular events, etc. [28], this should be considered when evaluating a patient with COVID-19. There is a controversy regarding whether the presence of neurotological symptoms justifies the use of chest CT scan to rule out clinically silent lung disease [11]; interestingly, in our study, there was no significant relationship between positive CT scan and neurotological symptoms (p = 0.407), which leads us to the conclusion that nervous system involvement is not synonymous of pulmonary involvement.

Otorhinolaryngological symptoms and the neurotologic profile

Loss of smell and taste have been described as clinical features of COVID-19 that persist even after the disease is resolved [29, 30]. In our study, almost half of the surveyed population presented anosmia (45%), which is similar to previous studies [29-31]. This clinical symptom is more frequent in patients with mild-moderate disease and it has also been considered the strongest predictor of positivity. In our study, loss of smell was associated with a neurotological profile (87.2% vs. 61.2%, p = 0.002).

Probably the invasion of one cranial nerve such as olfaction, could lead to a similar invasion of other cranial nerves (cochlear and/or vestibular), but this remains unknown [19, 20].

This study showed an increased prevalence of taste disorders (ageusia/hypogeusia of 58.4%) compared to other studies (38.3-45%) [29]. Moreover, in our study, there was an association with a neurotological profile and taste disorders (81.6% vs. 53.8%, p = 0.002).

The main limitation of our study is that it merely relies on a survey; therefore, more prospective studies are necessary to expand our knowledge on this disease. Our research group decided to perform a survey on health care workers because it minimizes bias, since health care workers are more aware of the clinical manifestations of this disease than the general population.

This is a study that explores the neurotologic symptoms of COVID-19 population and could probably reveal, by the creation of a neurotologic profile, the clinical features associated with a neurotologic presentation.

COVID-19 positive health care workers presented with scant but diverse neurotologic manifestations. The main clinical features associated with neurotologic symptoms were asthenia, smell and taste disorders.

## Conclusions

The most common neurotological manifestations were vertigo, tinnitus and imbalance. Clinical features associated with a neurotologic profile of symptoms were asthenia, hyposmia and dysgeusia.

## References

[1] Ge H, Wang X, Yuan X (2020). The epidemiology and clinical information about COVID-19. Eur J Clin Microbiol Infect Dis.

[2] Román GC, Spencer PS, Reis J (2020). The neurology of COVID-19 revisited: a proposal from the Environmental Neurology Specialty Group of the World Federation of Neurology to implement international neurological registries. J Neurol Sci.

[3] Gu J, Korteweg C (2007). Pathology and pathogenesis of severe acute respiratory syndrome. Am J Pathol.

[4] Desforges M, Le Coupanec A, Stodola JK, Meessen-Pinard M, Talbot PJ (2014). Human coronaviruses: viral and cellular factors involved in neuroinvasiveness and neuropathogenesis. Virus Res.

[5] Baig AM, Khaleeq A, Ali U, Syeda H (2020). Evidence of the COVID-19 virus targeting the CNS: tissue distribution, host-virus interaction, and proposed neurotropic mechanisms. ACS Chem Neurosci.

[6] Almufarrij I, Uus K, Munro KJ (2020). Does coronavirus affect the audio-vestibular system? A rapid systematic review. Int J Audiol.

[7] Ozer F, Alkan O (2021). Simultaneous sudden hearing loss and peripheral facial paralysis in a patient with Covid-19 (PREPRINT). Ear Nose Throat J.

[8] Giannantonio S, Scorpecci A, Montemurri B, Marsella P (2021). Case of COVID-19-induced vestibular neuritis in a child. BMJ Case Rep.

[9] Fancello V, Hatzopoulos S, Corazzi V (2021). SARS-CoV-2 (COVID-19) and audio-vestibular disorders. Int J Immunopathol Pharmacol.

[10] Mustafa MW (2020). Audiological profile of asymptomatic Covid-19 PCR-positive cases. Am J Otolaryngol.

[11] Karimi-Galougahi M, Naeini AS, Raad N, Mikaniki N, Ghorbani J (2020). Vertigo and hearing loss during the COVID-19 pandemic - is there an association?. Acta Otorhinolaryngol Ital.

[12] Lima MA, Silva MT, Soares CN (2020). Peripheral facial nerve palsy associated with COVID-19. J Neurovirol.

[13] Islamoglu Y, Celik B, Kiris M (2021). Facial paralysis as the only symptom of COVID-19: a prospective study. Am J Otolaryngol.

[14] Viola P, Ralli M, Pisani D (2021). Tinnitus and equilibrium disorders in COVID-19 patients: preliminary results. Eur Arch Otorhinolaryngol.

[15] Celis-Aguilar E, Espinoza-Valdez A, Torres-Gerardo F, López ED (2021). Questionnaire of otolaryngologic and neurotologic symptoms of COVID-19 positive health care workers. figshare.

[16] Das G, Mukherjee N, Ghosh S (2020). Neurological insights of COVID-19 pandemic. ACS Chem Neurosci.

[17] Di Carlo DT, Montemurro N, Petrella G, Siciliano G, Ceravolo R, Perrini P (2021). Exploring the clinical association between neurological symptoms and COVID-19 pandemic outbreak: a systematic review of current literature. J Neurol.

[18] Fiani B, Covarrubias C, Desai A, Sekhon M, Jarrah R (2020). A contemporary review of neurological sequelae of COVID-19. Front Neurol.

[19] Li YC, Bai WZ, Hashikawa T (2020). The neuroinvasive potential of SARS-CoV2 may play a role in the respiratory failure of COVID-19 patients. J Med Virol.

[20] Bougakov D, Podell K, Goldberg E (2021). Multiple neuroinvasive pathways in COVID-19. Mol Neurobiol.

[21] Politi LS, Salsano E, Grimaldi M (2020). Magnetic resonance imaging alteration of the brain in a patient with coronavirus disease 2019 (COVID-19) and anosmia. JAMA Neurol.

[22] Özçelik Korkmaz M, Eğilmez OK, Özçelik MA, Güven M (2021). Otolaryngological manifestations of hospitalised patients with confirmed COVID-19 infection. Eur Arch Otorhinolaryngol.

[23] Mady OM, El-Ozairy HS, Wady EM (2021). Increased incidence of otitis externa in covid-19 patients. Am J Otolaryngol.

[24] Saniasiaya J, Kulasegarah J (2021). Dizziness and COVID-19. Ear Nose Throat J.

[25] Almufarrij I, Munro KJ (2021). One year on: an updated systematic review of SARS-CoV-2, COVID-19 and audio-vestibular symptoms. Int J Audiol.

[26] Gupta S, Jawanda MK, Taneja N, Taneja T (2021). A systematic review of Bell's Palsy as the only major neurological manifestation in COVID-19 patients. J Clin Neurosci.

[27] Egilmez OK, Gündoğan ME, Yılmaz MS, Güven M (2021). Can COVID-19 cause peripheral facial nerve palsy?. SN Compr Clin Med.

[28] Ahmad I, Rathore FA (2020). Neurological manifestations and complications of COVID-19: a literature review. J Clin Neurosci.

[29] Brann DH, Tsukahara T, Weinreb C (2020). Non-neuronal expression of SARS-CoV-2 entry genes in the olfactory system suggests mechanisms underlying COVID-19-associated anosmia. Sci Adv.

[30] Yan CH, Prajapati DP, Ritter ML, DeConde AS (2020). Persistent smell loss following undetectable SARS-CoV-2. Otolaryngol Head Neck Surg.

[31] (2021). RE: "Covid-19 in health-care workers: a living systematic review and meta-analysis of prevalence, risk factors, clinical characteristics, and outcomes". Am J Epidemiol.

